The article "Comprehensive Analysis of Differentially Expressed Circular RNAs in Patients with Senile Osteoporotic Vertebral Compression Fracture" was published in 2020. Journal: Biomed Res Int.

# Comprehensive Analysis of Differentially Expressed Circular RNAs in Patients with Senile Osteoporotic Vertebral Compression Fracture

**DOI:** 10.1155/2020/4951251

**Published:** 2020-10-01

**Authors:** Xiaocong Yao, Minbo Liu, Fang Jin, Zhongxin Zhu

**Affiliations:** ^1^Department of Osteoporosis Care and Control, The First People's Hospital of Xiaoshan District, Hangzhou, Zhejiang 311200, China; ^2^Institute of Orthopaedics and Traumatology of Zhejiang Chinese Medical University, Hangzhou, Zhejiang 310053, China

## Abstract

**Aim:**

Circular RNAs (circRNAs) have been found to contribute to the regulation of many diseases and are abundantly expressed in various organisms. The present study is aimed at systematically characterizing the circRNA expression profiles in patients with senile osteoporotic vertebral compression fracture (OVCF) and predicting the potential functions of the regulatory networks correlated with these differentially expressed circRNAs.

**Methods:**

The circRNA expression profile in patients with senile OVCF was explored by using RNA sequencing. The prediction of the enriched signaling pathways and circRNA-miRNA networks was conducted by bioinformatics analysis. Real-time quantitative PCR was used to validate the selected differentially expressed circRNAs from 20 patients with senile OVCF relative to 20 matched healthy controls.

**Results:**

A total of 884 differentially expressed circRNAs were identified, of which 554 were upregulated and 330 were downregulated. The top 15 signaling pathways associated with these differentially expressed circRNAs were predicted. The result of qRT-PCR of the selected circRNAs was consistent with RNA sequencing.

**Conclusions:**

CircRNAs are differentially expressed in patients with senile OVCF, which might contribute to the pathophysiological mechanism of senile osteoporosis.

## 1. Introduction

Osteoporosis has been the most common age-related bone disorder characterized by low bone mineral density (BMD) and deterioration of microarchitecture with increased bone fragility and subsequent susceptibility to fractures [1, 2]. Senior population with osteoporosis often suffers from a fragility fracture, which will remarkably influence their life quality and increase family economic burden [3]. With the aging of the population, this burden has been increasing drastically. In addition, every low-energy fracture is linked to a raised risk of a subsequent fracture, which indicates a high risk of poor outcomes, and this risk is higher in men than women in the elderly [4]. In spite of its severe harm, osteoporosis is normally asymptomatic clinically at the early stage, and it is always ignored until the first fragility fracture happens. Clinically, primary osteoporosis can be divided into postmenopausal osteoporosis and senile osteoporosis. Senile osteoporosis, a common age-related degenerative disease, is characterized by impaired bone formation principally with a low bone turnover state [5, 6], whereas postmenopausal osteoporosis is related to excessive bone absorption owing to estrogen deficiency [7]. Despite the advances in therapeutic strategies, the diagnosis of senile osteoporosis at an early stage and the poor prognosis remains challenging. Therefore, there is an urgent need for a better understanding of the pathogenesis of senile osteoporosis in order to identify novel biomarkers and to develop new treatment strategies for the prevention and treatment of senile osteoporosis.

The article "Comprehensive Analysis of Differentially Expressed Circular RNAs in Patients with Senile Osteoporotic Vertebral Compression Fracture" was published in 2020. Journal: Biomed Res Int.

Emerging evidences demonstrate that microRNAs (miRNAs) are essential for bone remodeling and regeneration through the posttranscriptional regulation of gene expression [8–10]. With the development of next-generation sequencing technology, more noncoding RNAs have been discovered. As a large class of noncoding RNAs, circular RNAs (circRNAs) have multiple biological properties, such as high conservation, widespread expression, specific expression, and high stability [11–13]. Furthermore, some studies have reported that circRNAs were involved in age-related disease and played important roles in many biological processes as miRNA sponges [14]. Nevertheless, information about circRNAs on senile osteoporosis is very limited.

In this study, we used RNA sequencing, a powerful and unbiased approach to identify and analyze the differences in expression profiles of circRNAs and their regulatory interaction networks in patients with senile osteoporotic vertebral compression fracture (OVCF). These findings may help elucidate the mechanism underlying senile osteoporosis development and uncover novel diagnostic biomarkers for senile osteoporosis.

## 2. Materials and Methods

### 2.1. Patients and Samples

This study was approved by the Ethics Committee of our hospital. Fresh peripheral blood and written informed consent were attained from patients with newly diagnosed senile OVCF and healthy volunteers receiving a regular physical examination at the same hospital. The diagnosis for senile OVCF was confirmed through magnetic resonance imaging, dual-energy X-ray absorptiometry, and the history of patients. To decrease sources of circRNA expression heterogeneity not connected with disease status, selected subjects were all male, with similar age and body mass index. 2 ml blood was collected in ethylenediaminetetraacetic acid (EDTA) tube and mixed with three volumes of RNASaferTM LS Reagent (Magen, Guangzhou, China), then stored at -80C for batch processing.

The article "Comprehensive Analysis of Differentially Expressed Circular RNAs in Patients with Senile Osteoporotic Vertebral Compression Fracture" was published in 2020. Journal: Biomed Res Int.

### 2.2. RNA Extraction and High-Throughput Sequencing Analysis

Total RNA was extracted by Hipure PX Blood RNA Mini Kit (Magen) according to the manufacturer's protocol. The concentration and integrity of the isolated RNA were evaluated with Qubit 3.0 Fluorometer (Invitrogen, Carlsbad, California) and Agilent 2100 Bioanalyzer (Applied Biosystems, Carlsbad, CA). High-throughput sequencing was performed by Illumina Hiseq Xten to determine circRNAs in patients with senile OVCF (*n* = 3) and the controls (*n* = 3).

### 2.3. Data Analysis

We used Bowtie2 version 2.1.0 to map the reads to the latest UCSC transcript set and RSEM v1.2.15 to estimate the gene expression levels. We performed TMM to normalize the gene expression. We used edgeR program to perform quantile normalization and subsequent data processing. We used STAR to map the reads to the genome. We used DCC to identify the circRNAs and estimate their expression. CircRNAs were considered differentially expressed according to *P* < 0.01 and absolute log fold change >2.

### 2.4. Bioinformatics Analysis

Gene ontology (GO), Kyoto Encyclopedia of Genes and Genomes (KEGG), and Reactome pathway analyses of the differentially expressed circRNAs were performed by clusterProfiler R package. The related target miRNAs of circRNAs were identified by miRanda (v3.3). The circRNA-miRNA-mRNA network was constructed by Cytoscape software (v3.7.1).

### 2.5. Real-Time Quantitative PCR (qRT- PCR)

We selected circ_0079449 and circ_0122913 to validate the expression by qRT-PCR in 20 pairs of blood tissues from senile OVCF patients and normal controls. The qRT-PCR was carried out by the Geneseed qPCR SYBR Green Master Mix on ABI 7500 system. We used glyceraldehyde 3-phosphate dehydrogenase (GAPDH) as the internal control. The relative gene expression levels were analyzed using 2^-*ΔΔ*ct^ method against GAPDH for normalization. The primer sequences were as follows: circ_0079449, forward: 5′-ATTACTCTGTCGAAGTTGAA-3′, reverse: 5′-ATCACATACAGCTTTTTGTT-3′; circ_0122913, forward: 5′-GTTGGAACATCATAAACGA-3′, reverse: 5′-TGATTTCAACTTGTTCTTCT-3′. Their splicing junction sites are shown in Figure 1(a). Statistical analysis was performed by SPSS 24.0 software with a significance level of *P* < 0.05.

## 3. Results

### 3.1. Expression Profiles of Differentially Expressed circRNAs

RNA sequencing was performed to identify circRNAs in peripheral blood in three patients with senile OVCF and three healthy controls. We discovered 884 differentially expressed circRNAs (554 upregulated and 330 downregulated). The variations in circRNA expression were demonstrated by scatter maps and volcano plots (Figures 2(a) and 2(b)). Hierarchical clustering heat map analysis presented a recognizable circRNA expression profile in these two groups (Figure 2(c)).

The article "Comprehensive Analysis of Differentially Expressed Circular RNAs in Patients with Senile Osteoporotic Vertebral Compression Fracture" was published in 2020. Journal: Biomed Res Int.

### 3.2. GO, KEGG, Reactome Analysis, and circRNA–miRNA Network Analysis

To explore the role of differentially expressed circRNAs, GO, KEGG, and Reactome analyses and circRNA–miRNA network analysis were performed. The top three GO terms in the biological process (BP) were “DNA replication, nuclear chromosome segregation, mitotic nuclear division”, and “peptidyl−serine phosphorylation, protein methylation, histone methylation” for upregulated and downregulated circRNAs, respectively. The top three GO terms in the cellular component (CC) were “chromosome, centromeric region, microtubule organizing center part, condensed chromosome”, and “ribonucleoprotein granule, nuclear transcription factor complex, cytoplasmic ribonucleoprotein granule” for upregulated and downregulated circRNAs, respectively. The top three GO terms in the molecular function (MF) were “histone binding, protein C−terminus binding, modification−dependent protein binding”, and “Ras guanyl−nucleotide exchange factor activity, phosphatidylinositol binding, histone methyltransferase activity” for upregulated and downregulated circRNAs, respectively.

The top 10 most enriched GO terms of the upregulated and downregulated circRNAs in BP, CC, and MF are shown in Figures 3(a) and 4(a), respectively. The top three KEGG pathways were “RNA transport, cell cycle, and Hippo signaling pathway”, and “MAPK signaling pathway, human T−cell leukemia virus 1 infection, and T cell receptor signaling pathway” for upregulated and downregulated circRNAs, respectively. The top three Reactome pathways were “M Phase, transcriptional regulation by TP53, and DNA repair”, and “chromatin organization, chromatin modifying enzymes, and regulation of TP53 activity” for upregulated and downregulated circRNAs, respectively. The top 15 KEGG and Reactome pathways related to the upregulated and downregulated circRNAs are shown in Figures 3(b), 3(c), 4(b) and 4(c), respectively. The circRNA–miRNA coexpression network analysis of these differentially expressed circRNAs is shown in Figure 5.

### 3.3. qRT-PCR Validation and circRNA-miRNA-mRNA Network of the Selected circRNAs

The result of qRT-PCR was consistent with the sequencing data and showed significant differences in expression for circ_0079449 and circ_0122913 (Figure 1(b)). Next, we showed the five miRNAs that most potentially bind to circ_0079449 or circ_0122913, and the top five target genes to each miRNA in the illustration (Figure 1(c)).

## 4. Discussion

In the present study, after strict filtering of approximately 180 million reads, we detected 76547 circRNAs, including 884 circRNAs that were differentially expressed between patients with senile OVCF and control individuals. Based on GO, KEGG, and Reactome analyses, the functions of differentially expressed circRNAs were enriched. Moreover, their regulatory interaction networks were constructed. These results will be beneficial in future investigations of the molecular mechanism associated with senile osteoporosis.

miRNA is one kind of most studied regulators in the bone remodeling process and likely to be the diagnostic biomarker for osteoporosis [15]. Previous studies revealed miRNAs might play critical roles in the development of osteoporosis. For example, Mäkitie et al. [16] found circulating miRNAs in serum reflected status of WNT1 mutation, which leads to skeletal pathologies. Zhang et al. [17] found that miRNA-9-5p was lowly expressed in peripheral blood of osteoporosis patients and promoted the occurrence and progression of osteoporosis through inhibiting osteogenesis and promoting adipogenesis via targeting Wnt3a. In addition, miRNA-based therapies have shown great potential to become novel approaches against osteoporosis and associated fractures [8]. As miRNA sponges, circRNAs can adsorb miRNAs and eliminate the inhibitory effects of miRNAs on their target genes, leading to upregulation of target genes [18]. Besides, circRNAs are more stable than linear RNA due to their closed-loop structure [19]. CircRNAs have been considered potentially promising blood biomarkers in some musculoskeletal-related disease [20–22]. However, information about circRNAs on osteoporosis is limited.

The article "Comprehensive Analysis of Differentially Expressed Circular RNAs in Patients with Senile Osteoporotic Vertebral Compression Fracture" was published in 2020. Journal: Biomed Res Int.

Zhao et al. [23] used chip microarray analysis to investigate circRNA expression in postmenopausal osteoporosis and healthy menopausal women. Their data identified 203 upregulated and 178 downregulated circRNAs and revealed circ_0001275 was a potential diagnostic biomarker according to qRT-PCR results. Huang et al. [24] performed microarray analysis and PCR validation, and their result showed that circ_0006873 and circ_0002060 were linked to the low BMD state. In our study, rather than investigating by microarray which could identify only thousands of circRNAs, we chose to sequence all circRNAs that were attained in blood samples from patients with newly diagnosed senile OVCF and healthy controls.

Even though we identified the differentially expressed circRNAs in patients with senile OVCF, the underlying mechanism is still poorly understood. The GO terms provide computable knowledge regarding the activities of gene products and have been good predictors of them [25]. KEGG is an integrated database for biological interpretation of genome sequences and widely used in the enrichment analysis [26]. Reactome is a knowledgebase of biomolecular pathways and can be combined with other databases [27, 28]. Therefore, we systematically predicted the circRNA-related functions and corresponding pathways in senile osteoporosis with GO, KEGG, and Reactome analyses. In the present study, we found several pathways in the enrichment analysis were associated with osteoporosis. These pathways include the mitogen-activated protein kinase (MAPK) signaling pathway, DNA damage, DNA repair, and Th17 cell differentiation. Previous studies reported that the MAPK signaling pathway plays important roles in bone metabolism [29–31]. Other pathways were also involved in the development of osteoporosis, such as DNA damage, DNA repair, and Th17 cell differentiation [32–35]. The results suggest that these circRNAs might play roles in regulating physiological processes of osteoporosis.

The article "Comprehensive Analysis of Differentially Expressed Circular RNAs in Patients with Senile Osteoporotic Vertebral Compression Fracture" was published in 2020. Journal: Biomed Res Int.

There are some limitations in this study. First, our patients were carefully selected. We chose male and age, BMI-matched subjects from a single center. Although this decreased heterogeneity for this initial study, it would limit the generalizability of our findings. Second, the sample of this study is small. Therefore, a larger number of clinical samples are needed to confirm our results. Furthermore, the mechanism and function of the differentially expressed circRNAs should be further verified by strict molecular biological experiments research and studied deeply in future work.

In summary, we reported the circRNA expression profile in patients with senile OVCF by RNA sequencing analyses. Their regulatory interaction networks were constructed based on the sequencing data. These original discoveries might provide some clues for the biological functions of circRNAs in the pathophysiological mechanism of senile osteoporosis.

## Figures and Tables

**Figure 1:** The qRT-PCR validation in the 20 paired blood samples from patients with senile OVCF compared with normal group and circRNA-miRNA-mRNA network prediction of circ_0079449 and circ_0122913. (a) The splicing junction sites of circ_0079449 and circ_0122913 were indicated by black arrow. (b) The relative expression of circ_0079449 and circ_0122913. (c) The top 5 miRNAs potentially regulated by circ_0079449 and circ_0122913, respectively, and top 5 target genes of each miRNA. OVCF, osteoporotic vertebral compression fracture.

**Figure 2:** Next-generation sequencing to identify the differences in expression profiles of circRNAs between the senile OVCF and control groups. (a, b) The volcano plot and scatter plot showed the dysregulated circRNAs. Green and red denote significantly downregulated circRNAs and upregulated circRNAs, respectively. (c) Hierarchical clustering heat map showes the circRNAs with altered expressions in senile OVCF samples compared with controls. Each column represents one sample and each row represents one circRNA. OVCF: osteoporotic vertebral compression fracture; circRNA: circular RNA.

The article "Comprehensive Analysis of Differentially Expressed Circular RNAs in Patients with Senile Osteoporotic Vertebral Compression Fracture" was published in 2020. Journal: Biomed Res Int.

**Figure 3:** GO, KEGG, and Reactome analyses of upregulated circRNAs. (a) Top 10 GO analysis to demonstrate the molecular functions of upregulated circRNAs (b) Top 15 significant enrichment KEGG pathways of upregulated circRNAs. (c) Top 15 significant enrichment Reactome pathways of upregulated circRNAs. GO: Gene Ontology; KEGG: Kyoto Encyclopedia of Genes and Genomes; circRNA: circular RNA.

**Figure 4:** GO, KEGG, and Reactome analyses of downregulated circRNAs. (a) Top 10 GO analysis to demonstrate the molecular functions of upregulated circRNAs (b) Top 15 significant enrichment KEGG pathways of downregulated circRNAs. (c) Top 15 significant enrichment Reactome pathways of downregulated circRNAs. GO: Gene Ontology; KEGG: Kyoto Encyclopedia of Genes and Genomes; circRNA: circular RNA.

**Figure 5:** The potential regulatory network of circRNA-miRNA interactions in peripheral blood from patients with senile OVCF. Red triangle node and blue triangle node represent upregulated and downregulated circRNAs,respectively. Blue circular node represents miRNAs. OVCF: osteoporotic vertebral compression fracture; circRNA: circular RNA; miRNA: microRNA.

## Data Availability

The RNA-seq data have been uploaded to NCBI SRA database (Number: PRJNA562388).

## References

[1] Kanis J. A., McCloskey E. V., Johansson H., Oden A., Melton L. J., Khaltaev N. (2008). A reference standard for the description of osteoporosis. *Bone*.

[2] Jacobs E., Senden R., McCrum C., van Rhijn L. W., Meijer K., Willems P. C. (2019). Effect of a semirigid thoracolumbar orthosis on gait and sagittal alignment in patients with an osteoporotic vertebral compression fracture. *Clinical Interventions in Aging*.

[3] Mohd-Tahir N. A., Li S. C. (2017). Economic burden of osteoporosis-related hip fracture in Asia: a systematic review. *Osteoporosis International*.

[4] Center J. R. (2017). Fracture burden: what two and a half decades of Dubbo osteoporosis epidemiology study data reveal about clinical outcomes of osteoporosis. *Current Osteoporosis Reports*.

[5] Xie Y., Gao Y., Zhang L., Chen Y., Ge W., Tang P. (2018). Involvement of serum-derived exosomes of elderly patients with bone loss in failure of bone remodeling via alteration of exosomal bone-related proteins. *Aging Cell*.

[6] Farr J. N., Xu M., Weivoda M. M. (2017). Targeting cellular senescence prevents age-related bone loss in mice. *Nature Medicine*.

The article "Comprehensive Analysis of Differentially Expressed Circular RNAs in Patients with Senile Osteoporotic Vertebral Compression Fracture" was published in 2020. Journal: Biomed Res Int.

[7] Kiernan J., Davies J. E., Stanford W. L. (2017). Concise review: musculoskeletal stem cells to treat age-related osteoporosis. *Stem Cells Translational Medicine*.

[8] Sun X., Guo Q., Wei W., Robertson S., Yuan Y., Luo X. (2019). Current progress on MicroRNA-Based gene delivery in the treatment of osteoporosis and osteoporotic fracture. *International Journal of Endocrinology*.

[9] Zhao W., Shen G., Ren H. (2018). Therapeutic potential of microRNAs in osteoporosis function by regulating the biology of cells related to bone homeostasis. *Journal of Cellular Physiology*.

[10] Feng Q., Zheng S., Zheng J. (2018). The emerging role of microRNAs in bone remodeling and its therapeutic implications for osteoporosis. *Bioscience Reports*.

[11] Yao R., Zou H., Liao W. (2018). Prospect of circular RNA in hepatocellular carcinoma: a novel potential biomarker and therapeutic target. *Frontiers in Oncology*.

[12] Chen L. L. (2016). The biogenesis and emerging roles of circular RNAs. *Nature Reviews. Molecular Cell Biology*.

[13] Jeck W. R., Sorrentino J. A., Wang K. (2013). Circular RNAs are abundant, conserved, and associated with ALU repeats. *RNA*.

[14] Cai H., Li Y., Niringiyumukiza J. D., Su P., Xiang W. (2019). Circular RNA involvement in aging: an emerging player with great potential. *Mechanisms of Ageing and Development*.

[15] Materozzi M., Merlotti D., Gennari L., Bianciardi S. (2018). The potential role of miRNAs as new biomarkers for osteoporosis. *International Journal of Endocrinology*.

[16] Makitie R. E., Hackl M., Niinimaki R., Kakko S., Grillari J., Makitie O. (2018). Altered microRNA profile in osteoporosis caused by impaired WNT signaling. *The Journal of Clinical Endocrinology and Metabolism*.

[17] Zhang H. G., Wang X. B., Zhao H., Zhou C. N. (2019). MicroRNA-9-5p promotes osteoporosis development through inhibiting osteogenesis and promoting adipogenesis via targeting Wnt3a. *European Review for Medical and Pharmacological Sciences*.

[18] Hansen T. B., Jensen T. I., Clausen B. H. (2013). Natural RNA circles function as efficient microRNA sponges. *Nature*.

[19] Li X., Yang L., Chen L. L. (2018). The biogenesis, functions, and challenges of circular RNAs. *Molecular Cell*.

[20] Dolinar A., Koritnik B., Glavač D., Ravnik-Glavač M. (2019). Circular RNAs as potential blood biomarkers in amyotrophic lateral sclerosis. *Molecular Neurobiology*.

[21] Luo Q., Zhang L., Li X. (2018). Identification of circular RNAs hsa_circ_0044235 in peripheral blood as novel biomarkers for rheumatoid arthritis. *Clinical and Experimental Immunology*.

The article "Comprehensive Analysis of Differentially Expressed Circular RNAs in Patients with Senile Osteoporotic Vertebral Compression Fracture" was published in 2020. Journal: Biomed Res Int.

[22] Iparraguirre L., Munoz-Culla M., Prada-Luengo I., Castillo-Trivino T., Olascoaga J., Otaegui D. (2017). Circular RNA profiling reveals that circular RNAs from *ANXA*2 can be used as new biomarkers for multiple sclerosis. *Human Molecular Genetics*.

[23] Zhao K., Zhao Q., Guo Z. (2018). Hsa_Circ_0001275: a potential novel diagnostic biomarker for postmenopausal osteoporosis. *Cellular Physiology and Biochemistry*.

[24] Huang Y., Xie J., Li E. (2019). Comprehensive circular RNA profiling reveals circ_0002060 as a potential diagnostic biomarkers for osteoporosis. *Journal of Cellular Biochemistry*.

[25] The Gene Ontology Consortium (2019). The Gene Ontology Resource: 20 years and still GOing strong. *Nucleic Acids Research*.

[26] Kanehisa M., Sato Y., Furumichi M., Morishima K., Tanabe M. (2019). New approach for understanding genome variations in KEGG. *Nucleic Acids Research*.

[27] Fabregat A., Korninger F., Viteri G. (2018). Reactome graph database: efficient access to complex pathway data. *PLoS Computational Biology*.

[28] Bauer-Mehren A., Furlong L. I., Sanz F. (2009). Pathway databases and tools for their exploitation: benefits, current limitations and challenges. *Molecular Systems Biology*.

[29] Wu H., Hu B., Zhou X. (2018). Artemether attenuates LPS-induced inflammatory bone loss by inhibiting osteoclastogenesis and bone resorption via suppression of MAPK signaling pathway. *Cell Death & Disease*.

[30] Thouverey C., Caverzasio J. (2015). Focus on the p38 MAPK signaling pathway in bone development and maintenance. *BoneKEy reports*.

[31] Zheng S., Wang Y. B., Yang Y. L. (2019). LncRNA MALAT1 inhibits osteogenic differentiation of mesenchymal stem cells in osteoporosis rats through MAPK signaling pathway. *European Review for Medical and Pharmacological Sciences*.

[32] Ghayor C., Weber F. E. (2016). Epigenetic regulation of bone remodeling and its impacts in osteoporosis. *International Journal of Molecular Sciences*.

[33] Wu X., Li J., Zhang H., Wang H., Yin G., Miao D. (2017). Pyrroloquinoline quinone prevents testosterone deficiency-induced osteoporosis by stimulating osteoblastic bone formation and inhibiting osteoclastic bone resorption. *American Journal of Translational Research*.

[34] You L., Chen L., Pan L., Peng Y., Chen J. (2018). SOST gene inhibits osteogenesis from adipose-derived mesenchymal stem cells by inducing Th17 cell differentiation. *Cellular Physiology and Biochemistry*.

[35] Zhao R. (2013). Immune regulation of bone loss by Th17 cells in oestrogen-deficient osteoporosis. *European Journal of Clinical Investigation*.

